The article "Unique RNA signature of different lesion types in the brain white matter in progressive multiple sclerosis" was retracted in 2019. Reasons: errors in the data; errors in the analysis; errors in the results or conclusions.

# Unique RNA signature of different lesion types in the brain white matter in progressive multiple sclerosis

**DOI:** 10.1186/s40478-019-0709-3

**Published:** 2019-04-25

**Authors:** Maria L. Elkjaer, Tobias Frisch, Richard Reynolds, Tim Kacprowski, Mark Burton, Torben A. Kruse, Mads Thomassen, Jan Baumbach, Zsolt Illes

**Affiliations:** 1 Department of Neurology, Odense University Hospital, J.B. Winslowsvej 4, DK-5000 Odense, Denmark; 2 Institute of Clinical Research, BRIDGE, University of Southern Denmark, Odense, Denmark; 3 Institute of Molecular Medicine, University of Southern Denmark, Odense, Denmark; 4 Department of Mathematics and Computer Science, University of Southern Denmark, Odense, Denmark; 5 Division of Brain Science, Imperial College, London, UK; 6 Research Group Computational Systems Medicine, Chair of Experimental Bioinformatics, TUM School of Life Sciences Weihenstephan, Technical University of Munich, Munich, Germany; 7 Department of Clinical Genetics, Odense University Hospital, Odense, Denmark; 8 Chair of Experimental Bioinformatics, TUM School of Life Sciences Weihenstephan, Technical University of Munich, Munich, Germany

**Keywords:** Multiple sclerosis brain lesions, Next-generation RNA sequencing, TGF-beta, Chitinase-3-like protein-1, CD26/DPP4

## Abstract

The heterogeneity of multiple sclerosis is reflected by dynamic changes of different lesion types in the brain white matter (WM). To identify potential drivers of this process, we RNA-sequenced 73 WM areas from patients with progressive MS (PMS) and 25 control WM. Lesion endophenotypes were described by a computational systems medicine analysis combined with RNAscope, immunohistochemistry, and immunofluorescence. The signature of the normal-appearing WM (NAWM) was more similar to control WM than to lesions: one of the six upregulated genes in NAWM was CD26/DPP4 expressed by microglia. Chronic active lesions that become prominent in PMS had a signature that were different from all other lesion types, and were differentiated from them by two clusters of 62 differentially expressed genes (DEGs). An upcoming MS biomarker, CHI3L1 was among the top ten upregulated genes in chronic active lesions expressed by astrocytes in the rim. TGFβ-R2 was the central hub in a remyelination-related protein interaction network, and was expressed there by astrocytes. We used de novo networks enriched by unique DEGs to determine lesion-specific pathway regulation, i.e. cellular trafficking and activation in active lesions; healing and immune responses in remyelinating lesions characterized by the most heterogeneous immunoglobulin gene expression; coagulation and ion balance in inactive lesions; and metabolic changes in chronic active lesions. Because we found inverse differential regulation of particular genes among different lesion types, our data emphasize that omics related to MS lesions should be interpreted in the context of lesion pathology. Our data indicate that the impact of molecular pathways is substantially changing as different lesions develop. This was also reflected by the high number of unique DEGs that were more common than shared signatures. A special microglia subset characterized by CD26 may play a role in early lesion development, while astrocyte-derived TGFβ-R2 and TGFβ pathways may be drivers of repair in contrast to chronic tissue damage. The highly specific mechanistic signature of chronic active lesions indicates that as these lesions develop in PMS, the molecular changes are substantially skewed: the unique mitochondrial/metabolic changes and specific downregulation of molecules involved in tissue repair may reflect a stage of exhaustion.

The article "Unique RNA signature of different lesion types in the brain white matter in progressive multiple sclerosis" was retracted in 2019. Reasons: errors in the data; errors in the analysis; errors in the results or conclusions.

**Electronic supplementary material:**

The online version of this article (10.1186/s40478-019-0709-3) contains supplementary material, which is available to authorized users.

## Introduction

Multiple sclerosis (MS) is a chronic inflammatory, demyelinating and neurodegenerative disease of the CNS. Without treatment, a secondary progressive course (SPMS) develops in about half of the patients [60]. Neuroimaging, treatment responses and pathology all show differences between the early and late phase of MS, indicating that disease mechanisms change during the natural course [28]. Therefore, modern systems medicine approaches may help to increase our understanding of MS progression and to find novel, mechanistic treatment targets.

Inflammatory demyelination affects osmotic homeostasis, energy coupling with oligodendrocytes, and contributes to glutamate excitotoxicity, axonal damage and fibrillary gliosis that may inhibit remyelination [21, 45, 46]. Key elements of the degenerative process are chronic oxidative injury [26], accumulation of mitochondrial damage resulting in chronic cell stress and imbalance of ionic homeostasis [13, 55], microglia activation, and age-related iron accumulation in the brain [57]. As the disease progresses, diffuse changes can be observed in the normal appearing white and grey matter (NAWM, NAGM), and B cell follicle-like cellular aggregates contribute to subpial cortical lesions [44, 46, 54, 68].

WM lesions are inherent characteristics of MS from the early phase, and both quantitative and qualitative changes in the WM can be observed as the disease progresses: microglia activation in the NAWM [20], increasing number of chronic active lesions, and decreasing number of remyelinating lesions [17, 66]. B cells are also present in active WM lesions in progressive MS, and the number of plasma cells is higher in lesions from progressive MS compared to acute MS [22, 53].

The article "Unique RNA signature of different lesion types in the brain white matter in progressive multiple sclerosis" was retracted in 2019. Reasons: errors in the data; errors in the analysis; errors in the results or conclusions.

The lesion evolution and fate in the WM can be classified into distinct groups based on the distribution and density of inflammatory cells and myelin loss [68]. During lesion evolution, active lesions develop from the NAWM and are characterized by myelin breakdown and massive infiltration by macrophages and activated microglia. Lesions may remyelinate [51], and partially remyelinated axons and activated microglia are seen [68]. Lesions can develop into inactive lesions with sharply demarcated hypocellular area of demyelination and axonal degeneration with little to no inflammatory activity [23, 68]. As the disease progresses, the number of chronic active (smoldering, slowly expanding, mixed active/inactive) lesions with a hypocellular demyelinated core and a rim of activated glia increases [23, 41, 51]. The number of chronic active lesions inversely correlates with the proportion of remyelinating lesions, and patients with more severe disease have a higher proportion of such lesions [51].

The molecular mechanisms driving the development and evolution of the different cellular MS endophenotypes are largely unknown. To identify dominant pathways of lesion genesis, unbiased omics investigation of precisely defined and microdissected lesions at these different stages of lesion formation and their comparison to controls is required. We address this need by generating and analyzing the first map of the transcriptional landscape of lesion evolution and fate in progressive MS brain by next-generation RNA sequencing to identify key pathways, molecules and their cellular source (Fig. 1). With our comprehensive transcriptomics data, we have been able to extract mechanistic signatures that differentiate between lesions. We identified lesion-specific protein complex networks by using de novo network enrichment. We further validated the differential expression of key molecules and examined their cellular source by RNAscope, immunohistochemistry, and by immunofluorescence. This specific selection and validation of mechanistic signatures in different lesion types emphasize the value of precision in the characterization of the diverse phenotype of lesions, when understanding the complex and heterogeneous pathogenesis of MS.

**Fig. 1:** Outline of the systems medicine approach to identify mechanistic MS lesion type drivers. Using RNAseq we analysed the transcriptome of normal-appearing white matter (NAWM), and lesion evolution/fate (active, inactive, chronic active, remyelinating) in the white matter (WM) of patients with progressive MS. We performed a comprehensive computational data analysis – from differential expression to de novo network enrichment – and examined selected molecules of interest by a combination of RNAscope, immunohistochemistry and immunofluorescence to confirm their cellular source and protein expression levels

The article "Unique RNA signature of different lesion types in the brain white matter in progressive multiple sclerosis" was retracted in 2019. Reasons: errors in the data; errors in the analysis; errors in the results or conclusions.

## Materials and methods

### Human postmortem brain tissue

MS and control tissue samples were supplied by the UK Multiple Sclerosis Tissue Bank (UK Multicentre Research Ethics Committee, MREC/02/2/39), funded by the Multiple Sclerosis Society of Great Britain and Northern Ireland (registered charity 207,495). A total of 73 snap-frozen tissue blocks from ten progressive MS patients and 25 blocks from five donors without neurological disease were chosen. The death-tissue preservation interval was between 8 and 30 h. Clinical data are summarized in Additional file 1: Table S1.

Lesion classification, antibodies and RNAScope are described in Additional file 2 and Additional file 3: Figure S1.

### RNA extraction from specific histological brain areas

The brain fields of interest were manually microdissected under a magnifying glass in a cryostat. The amount of collected tissue ranged between 10 and 100 mg/sample depending on the lesion size and thickness. A total of 25 WM control areas, 19 NAWM, 6 remyelinating, 18 active, 13 inactive and 17 chronic active lesions were harvested. Total RNA were isolated from the frozen brain samples according to the manufacturer’s instruction (miRNeasy Mini Kit, Qiagen) including DNAse I treatment. RNA concentration was measured using NanoDrop spectrophotometer ND-1000 (Thermo Scientific), and the integrity of RNA (RIN) was measured by using the Bioanalyzer 2100 (Agilent Technologies). RNA integrity was good quality (RIN 6 ± 1.7) among the samples. The fragmentation time and cleanup steps during library preparation have been adapted for each sample based on the RIN value.

### Next-generation sequencing

One μg of RNA per sample was processed to remove ribosomal RNA followed by library preparation for RNA sequencing using TruSeq Stranded Total RNA Library Prep Kit with Ribo-Zero Human/Mouse/Rat Set (Illumina). Pooled indexed libraries were loaded into flow cell followed by 2 × 80 bp paired-end sequencing on an Illumina NextSeq550.

### Raw data analysis and quality control

Demultiplexing was carried out with Casava software (IIlumina) configured to allow one mismatch during the identification of the indexes. Data were filtered with Trimmomatic [9] (TRIM:2:30:10 LEADING:20 TRAILING:20 SLIDING:4:20 TRAILING:20 MIN:17). Filtered transcripts were aligned against the human reference genome from UCSC [38] (GRCh38/hg38) with STAR 2.5.3a [14] using default mode/parameters and counted using HTSeq-count [5] using strict mode.

The article "Unique RNA signature of different lesion types in the brain white matter in progressive multiple sclerosis" was retracted in 2019. Reasons: errors in the data; errors in the analysis; errors in the results or conclusions.

### Statistical analysis

Differentially Expressed Genes (DEGs) between different lesion types vs. control WM were identified with the edgeR package (3.8) [70]. The generalized linear model used for our analysis adjusted for library size and biological replicates (same lesion type//same sample//from same patient). Furthermore, we corrected for age and sex of the patients. Genes that were lowly expressed were excluded following the edgeR userGuide. Therefore, genes were expected to be presented with more than two counts per million (CPM) in at least as many samples as present in the smallest lesion group. Adjusted *P* value filtering using the procedure of Benjamini and Hochberg was used to identify genes significantly differently expressed between MS brain areas and control brain areas.

### Volcano plots, heatmaps and pathways

Volcano plots and heatmaps were created in R studio, and Venn diagrams were produced using an online tool at http://bioinformatics.psb.ugent.be/webtools/Venn/. Predefined pathways were identified by importing the DEGs to Reactome [19], and enriched gene clusters of all detected genes were extracted from Gene Set Enrichment Analysis (GSEA) [77]. Raw pre-processed transcripts were also analysed by Ingenuity Pathway Analysis. KeyPathwayMiner [3, 4] was used to conduct *de-novo* network enrichment analyses. The biological network was extracted from the Integrated Interactions Database (IID) [40] restricted to only brain specific interactions based on evidence type: experimental detection, orthology or prediction. Hubs were selected based on the highest betweenness centrality value.

### Data availability

All data is deposited and can be post-analyzed online at “msatlas.dk”.

## Results

### Comparison of the WM transcriptome between MS and control

We defined significant differentially expressed genes (DEGs) with FDR < 0.05 compared to control WM.

First, we compared the transcriptome of the global MS tissue (NAWM and lesions) to control WM tissue: out of 18,722 detected genes, 4223 were DEGs. Around the same number of genes were detected, when individual lesion types were compared to control WM (Additional file 4: Table S2). More DEGs with fold change (log_2_FC > 1/<− 1, FDR < 0.05) were upregulated (*n* = 375) than downregulated (*n* = 109) in the MS WM transcriptome landscape (Fig. 2a).

**Fig. 2:** Change in gene expression profile during the evolution and fate of WM lesions in progressive MS. **a** Visualization of the transcriptional landscape of genes (*n* = 18,722) detected between MS and non-MS (dots in graph); significantly regulated (FDR < 0.05) genes are indicated in bright red and orange, where orange indicates log_2_FC > 1 or < − 1. **b** The Venn diagram represents the number of overlapping and lesion-specific differentially expressed genes (FDR < 0.05) between white matter (WM) lesion types (active, inactive, remyelinating, chronic active) compared to control WM tissue. FDR: false discovery rate; FC: fold change

We then compared DEGs between each lesion type in order to identify common and uniquely expressed genes (Fig. 2b). The lesion types had 260 DEGs in common, among them genes encoding for cytokines, chemokines, complement factors (e.g. *IL7R, IL15, TNFAIP8, CXCL12, CFI*) (data not shown). A high number of DEGs, 2415 were uniquely expressed, and therefore we focused on these differences in transcriptome signatures.

The article "Unique RNA signature of different lesion types in the brain white matter in progressive multiple sclerosis" was retracted in 2019. Reasons: errors in the data; errors in the analysis; errors in the results or conclusions.

To examine molecular processes, DEGs for each lesion type were uploaded to KEGG and GSEA, and the enriched pathways were extracted. We detected 26 and 33 shared pathways from KEGG and GSEA, respectively, such as the TNF signaling pathway, cytokine-cytokine receptor interaction, natural killer cell mediated cytotoxicity, T cell specific pathways and metabolic pathways (Additional file 5: Table S3). Furthermore, we detected significant enrichment of metabolic gene clusters and pathways in the control WM compared to the global MS-WM tissue, and some were uniquely represented only in the control WM suggesting a metabolic failure in the MS brain. We therefore examined the top 100 up- and downregulated DEGs related to oxidative stress, hypoxia and metabolic changes. The highest number of such dysregulated genes were found in chronic active lesions. In addition, while active, inactive and remyelinating lesions shared several of these DEGs (e.g. upregulated mitochondrial humanins and downregulated COX subunit), all the DEGs related to oxidative stress, hypoxia and metabolic changes in the chronic active lesions were unique (e.g. several mitochondrial genes) (Additional file 6: Table S4). Genes expressed in different lesion types were also analyzed by IPA. Based on significant up- and downregulated DEGs from the active lesions, IPA correctly identified the samples as originating from brain lesions, which supports the validity of the identified gene expression signatures (Additional file 7: Figure S2).

### Transcriptome signature of the normal-appearing with matter

To address changes before the evolution of lesions, we examined all DEGs in NAWM and examined if they remained differentially regulated as an active lesion develops. In the NAWM, we detected 6 upregulated and 16 downregulated DEGs (Fig. 3a) involved in angiogenesis (*VEGFA, ADM*), pro- and anti-inflammatory responses (*ATF3, SLC7A2*), cellular growth (*PIWIL2, SFRP2*) or hypoxia related conditions (*MT1M, DDIT4, PPP1r3C*). Out of these 22 genes, 13 genes were also significantly expressed in active lesions (Fig. 3b), while the 9 other were not.

The article "Unique RNA signature of different lesion types in the brain white matter in progressive multiple sclerosis" was retracted in 2019. Reasons: errors in the data; errors in the analysis; errors in the results or conclusions.

**Fig. 3:** Molecular signature of NAWM and CD26/DPP4 expression **a** Significant differentially expressed genes (DEGs, FDR < 0.05) in the normal-appearing white matter (NAWM) compared to control white matter (WM). **b** Expression of significant differentially expressed genes in the NAWM that remained significantly expressed in active lesions. **c** The protein expression of *CD26/DPP4* in the NAWM. *Lower panel:* co-localization of CD26/DPP4 with IBA1 in the NAWM. **d** Expression of CD26/DPP4 in an active lesion. FDR: false discovery rate; WM: white matter

### CD26/DPP4 expression by microglia in the normal-appearing with matter

Among the 6 upregulated DEGs in the NAWM, and among the 4 DEGs that remained upregulated in active lesions, we found *CD26/DPP4* encoding for dipeptidylpeptidase 4 (CD26, DPP4) that has previously been identified in NAWM by RNA-seq and DNA methylation analysis [32]. We confirmed the protein expression of CD26 in the NAWM, and its absence in control WM by immunohistochemistry (Fig. 3c). The morphology of cells expressing CD26 in NAWM indicated microglia, and CD26 co-localized with IBA1 (Fig. 3c). In the active lesions, CD26 was expressed by infiltrating lymphocytes or monocytes rather than microglia (Fig. 3d).

### The unique molecular signature of chronic active lesions

To identify unique transcriptome changes in different lesion types, and generate the molecular signatures of WM lesion types in progressive MS, we first selected the DEGs for each lesion type compared to control (FDR < 0.05). For each of these selected DEGs, we then calculated the fold-changes between the different lesions types, and kept only those for which we found at least three-times differential regulation for at least one pair of lesions types (Fig. 4).

**Fig. 4:** Transcriptome signature of lesion evolution and fate in progressive MS. Heatmap showing differential expression of genes (DEGs) in different white matter lesion types compared to control white matter (FDR < 0.05) with a selection of the DEGs with highest fold changes (log_2_FC > 1.5 for at least one pair of lesions types). FC: fold change, FDR: false discovery rate, NAWM: normal appearing white matter

We identified two distinct clusters of up- and downregulated 62 DEGs that clearly separated chronic active from all other lesion types by inverse regulation pattern, indicating again that chronic active is a very distinct lesion type. We also found that remyelinating and chronic active lesions had the most different DEGs pattern (Fig. 4). This characteristic signature of chronic active lesions included among others downregulated genes of repair/growth *(CD26/DPP4, IGF2, MERTK, MTRNR2L8, MTRNR2L12, FOXF1, FENDRR, PIK3R5, TNFRSF10D, GPNMB)* all upregulated in the other lesion types; and upregulated genes of angiogenesis/hypoxia condition *(ADM, HILPDA, VEGFA MiR210HG, COX5BP6, GPD1)*, inhibition of neural/axonal growth *(ZNF536, SEMA3B)*, collagen/tubulin production *(GALNT6, ADAMTST14, TBB4A)*, calcium channels *(TRPV6, STC2)* that were all downregulated in the other lesion types (Fig. 4).

The article "Unique RNA signature of different lesion types in the brain white matter in progressive multiple sclerosis" was retracted in 2019. Reasons: errors in the data; errors in the analysis; errors in the results or conclusions.

### CHI3L1, an astrocytic marker in the rim of chronic active lesions

We found that *CHI3L1,* the gene of an emerging CSF molecular marker [71] was among the top ten upregulated DEGs in chronic active lesions (FDR: 0.04 and log_2_FC: 1.74) **(**Additional file 8: Table S5), and was also uniquely upregulated in chronic active lesions **(**Fig. 5a**)**. In contrast, *CHI3L1* was downregulated in all the other lesion types **(**Fig. 5a**)**; it was among the top 10 downregulated DEGs in the MS brain tissue compared to control WM (FDR: 1.7 × 10^− 5^ and log_2_FC:-1.8), and among the top ten downregulated DEGs in NAWM and inactive lesions (Additional file 8: Table S5). By using immunohistochemistry, we verified the unique upregulation of CHI3L1 in chronic active lesions **(**Fig. 5b**).** The morphology of cells expressing CHI3L1 in chronic active lesions indicated astrocytes in the rim **(**Fig. 5c**)**. The astrocytic expression was confirmed by combined RNAscope and immunohistochemistry that co-localized *CHI3L1* and *GFAP/*GFAP at the chronic active rim in close proximity to MHCII expressing cells **(**Fig. 5d and e**)**; *CHI3L1* did not co-localize with microglia or macrophages (*IBA1* or MHCII) **(**Fig. 5f and g**)**.

**Fig. 5:** Chitinase-3-like protein 1 (CHI3L1) in the rim of chronic active lesions. **a** RNA expression of *CHI3L1* gene in each lesion type. log_2_FC (fold change) and significance (FDR, false discovery rate) is shown. **b** Protein expression of CHI3L1 protein in each lesion type. **c** Protein expression of CHI3L1 in the rim of chronic active lesion, and MOG staining defining the edge of the same lesion. **d** Protein expression of GFAP (brown) and RNA expression of *CHI3L1* (red) in same cells (combined immunohistochemistry and RNAscope). **e** Co-localized RNA expression of *GFAP* (red) with *CHI3L1* (green) by RNAscope. **f** Protein expression of MHCII (brown) and RNA expression of *CHI3L1* (red) in different cells close to each other at the rim of the lesion (combined immunohistochemistry and RNAscope). **g** RNA expression of *IBA1* (red) and *CHI3L1* (green) (RNAscope). WM: white matter, NAWM: normal appearing white matter. FDR: false discovery rate

The article "Unique RNA signature of different lesion types in the brain white matter in progressive multiple sclerosis" was retracted in 2019. Reasons: errors in the data; errors in the analysis; errors in the results or conclusions.

### Remyelination-specific de novo network, TGFβ-R2 and immunoglobulin signatures

Since we noticed that chronic active and remyelinating lesions differed the most on the heatmap of unique molecular signatures (Fig. 4), we extracted DEGs that were significantly upregulated (FDR < 0.05) in remyelinating while significantly downregulated in chronic active lesions. We identified 269 such genes, and next we examined their de novo enriched network based on protein-protein interactions. The biggest network contained 63 proteins of DEGs with 117 connections, which were all upregulated in remyelinating lesions while downregulated in chronic active lesions, and it suggested pathways of pro-and anti-inflammation (*IL7R, IL15, CXCL12, STAT6, DAB2, MERTK, A2M, CASP1, CASP4, ETS2, MICB, TRIM25/TYROBP*), cell growth (*EGF, GDF11, HIPK1/3, FOXF1, GPNMB, BMP2K, NFATC2, PGR, TNFAIP8, TNFSF10/TRAIL, ZEB1, ZNF217*), oxidative stress and DNA damage repair (*AMOT, CDC14A, GDP2, MAF, VEGFC, WWTR1*), and B cell related genes (*KLHL6, B4GALT1, IKZF1*). In this remyelination network, TGFβ-R2 was the central hub (Fig. 6a). Therefore, we examined gene expression of additional receptors of TGFβ and their ligands. Two of the three receptors and three out of five ligands were significantly (FDR < 0.05) upregulated in remyelinating lesions, but only *TGFBR2* was significantly downregulated in chronic active lesions (Fig. 6b). We also stained for TGFβ-R2 in remyelinating lesions, and the cell morphology of positive cells indicated astrocytes (Fig. 6c). By using RNAscope, we found *GFAP* and *TGFBR2* mRNA co-expressed in remyelinating lesions (Fig. 6d). Microglia did not express *TGFBR2*, as *IBA1* and *TGFBR2* were expressed in different cells far from each other (Fig. 6e).

**Fig. 6:** TGFβ-R2 in remyelinating versus chronic active lesions. **a** *De-novo* enriched protein-protein network of significant differentially regulated genes (DEGs, FDR < 0.05) that were downregulated in chronic active and upregulated in remyelinating lesions (63 nodes, 117 protein connections). **b** Genes of TGFβ receptors and ligands in different lesion types. Asterisk indicates significant changes (FDR < 0.05). **c** TGFβ-R2 protein expression in remyelinating lesions. **d** *TGFBR2* (green) RNA co-localizes with *GFAP* (red) RNA in remyelinating lesions by RNAscope. **e** *TGFBR2* (green) RNA do not co-localize with *IBA1* RNA by RNAscope. FDR: false discovery rate

We also noticed that immunoglobulin genes were present among the top 10 upregulated genes in the WM tissue of MS (Fig. 7a), especially in the active and remyelinating lesions (Additional file 8: Table S5). To examine the presence of B cells, we quantified CD20^+^ cells in active (*n* = 3) and remyelinating (*n* = 4) lesions each from different patients (*n* = 7), and found that they were mostly present in active lesions. We detected less B cells in remyelinating compared to active lesions, but none in chronic active lesions and in the NAWM **(**Fig. 7b and c)**.** This staining pattern correlated with the upregulated immunoglobulin transcripts in active and remyelinating lesions (log_2_FC: 10.16 in active and 12.66 in remyelinating lesions; FDR: 0.0001 in active and 0.01-8 × 10^− 11^ in remyelinating lesions). Remyelinating lesions had the most heterogenous upregulated transcripts for different variable regions **(**Fig. 7d**).** The gene of the plasma cell marker CD138 was uniquely upregulated in remyelinating lesions (log_2_FC:2.6, FDR: 0.0002).

The article "Unique RNA signature of different lesion types in the brain white matter in progressive multiple sclerosis" was retracted in 2019. Reasons: errors in the data; errors in the analysis; errors in the results or conclusions.

**Fig. 7:** Immunoglobulin signatures and B cells in WM lesions of patients with progressive MS. **a** Immunoglobulin transcripts among the top 10 upregulated DEGs (FDR < 0.05) in the global MS white matter (WM) tissue compared to control WM tissue. **b** Distribution of CD20^+^ cells within the different MS lesions used also for generating transcriptome signatures. **c** Number of CD20^+^ cells in active (*n* = 3) and remyelinating (*n* = 4) lesions, each lesion from different brains. The same brains and lesions were used for generating transcriptome signatures. Around 10 pictures per lesion in each patient were taken at magnification of 20x and the average cell number per lesion were calculated. Statistical difference between the CD20^+^ cells was calculated using the Mann-Whitney test. **d** Heatmap of immunoglobulin transcripts in the different lesion types. FDR: false discovery rate

### Unique de novo protein-protein networks of lesion evolution and fate

We also used another approach to examine lesion stage-specific gene expression. We extracted DEGs that were unique to specific lesions: 776 for active, 718 for remyelinating, 767 for inactive, and 154 for chronic active (Fig. 2b and Fig. 8a). By using KeyPathwayMiner we mapped each of these gene set to a brain specific protein-protein network, and retrieved the biggest de novo subnetwork with hubs for each lesion type (Fig. 8b). In the active lesion-specific biggest network, DEGs and hubs were related to immune recruitment (*ICAM1, CCR1, CD4, C5RA1*) and activation (*HLA-DPB1, HLA-DOA, HLA-DQA1, CD74, IL13RA1*). The remyelinating lesion-specific network contained DEGs and hubs related to tissue recovery/cellular growth (*PDGFRA*, *CNTNAP2, TNR, EPS15, ANLN, BMP4, KDR*) and immune responses (*CD3E, CD8A, IL1RAPL1, FCRL5, TNFAIP6*). The chronic active lesion-specific network included DEGs and hubs related to metabolic changes (*CDH2, PPARGC1A, DYRK1A*) and the major hubs were *IKBKG* coding for the NEMO protein and *CDH2* encoding for cadherin N. The inactive lesion-specific network DEGs and hubs were related to homeostatic control (*DNAJB1, GPX4, SLC4A4, SLC30A3, SLC17A7*) (Fig. 8b).

The article "Unique RNA signature of different lesion types in the brain white matter in progressive multiple sclerosis" was retracted in 2019. Reasons: errors in the data; errors in the analysis; errors in the results or conclusions.

**Fig. 8:** Lesion specific signatures and their biggest de novo network enrichment. **a** The heatmap indicates all differentially expressed genes (DEGs, FDR < 0.05) uniquely expressed in each lesion type (vertical lines). **b** By using KeyPathwayMiner, we retrieved the biggest de novo network from each of the lesion-specific gene list indicated on Fig. 8a: 56 nodes (log_2_FC > 1) (k = 0) in active; 59 nodes (log_2_FC > 1) (k = 0) in remyelinating; 31 nodes (k = 2, TB53, UBC) in chronic active; and 26 nodes (log_2_FC > 1), (k = 2, HEL2, UBC) in inactive lesions. k = exception nodes, genes not differentially expressed; UBC = ubiquitin C; TB53 = Tumor Suppressor P53; HEL2 = E3 ubiquitin-protein ligase/14–3-3 epsilon. More intensive colour indicates higher betweenness centrality of hubs. FC = fold change; FDR = false discovery rate

## Discussion

We introduce the first mechanistical investigation of transcriptome signatures of lesion evolution and fate in the WM of patients with progressive MS across all major WM lesion types: NAWM, active, inactive, chronic active and remyelinating lesions (compared to control WM). One study applied next generation RNA sequencing to examine gene expression in the NAWM [33], and a very recent work examined oligodendrocyte nuclei signatures in MS lesions [34]. We controlled for confounders using generalized mixed effect linear models considering age, sex and multiple samples of the same patient. We corrected all results for multiple testing with a target FDR value < 0.05 to use a conservative statistical estimation of gene expression changes. We still detected a high number of differently expressed genes in different lesion types (compared to the control samples). Most of these DEGs with high fold change were upregulated in the MS tissue. We then, for the first time, interrogated the human interactome for sub-networks that putatively drive MS lesion evolution mechanistically.

### Inverse expression of common genes in different lesion types

The lesions had 260 common DEGs (FDR < 0.05) (Fig. 2), but their direction of regulation changed depending on lesion type. For example, the transcript of the MS risk gene *IL7R* was significantly upregulated in active, inactive and remyelinating lesions, while significantly downregulated in the chronic active lesions, and was not detected in the NAWM. About ten times higher number of genes was uniquely expressed in particular lesion types, suggesting that there are significant transcriptional changes during lesion evolution that contribute to diverse molecular mechanisms related to the stage of the lesion. Therefore, it may be crucial to relate omics data in the MS brain to specific lesion types instead of subsuming all different lesions types as diseased tissue. Otherwise interpretation about up- or downregulation of individual molecules may be misleading, and disregard important changes in lesion evolution and fate.

The article "Unique RNA signature of different lesion types in the brain white matter in progressive multiple sclerosis" was retracted in 2019. Reasons: errors in the data; errors in the analysis; errors in the results or conclusions.

### Dipeptidylpeptidase IV (CD26/DPP4) expressed by microglia in the NAWM

We found that the transcriptome signature of NAWM resembled more to the control WM than to the transcription signature of any lesion types. Most of the 22 DEGs in NAWM were related to angiogenesis, pro- and anti-inflammation, hypoxia and cellular growth/differentiation indicating hypoxia and low-level inflammation before lesion evolution.

Out of the 22 DEGs of NAWM, 13 genes had the same expression pattern in active lesions (FDR < 0.05), suggesting that these could be pathogenic drivers for lesion evolution. One of these shared DEGs, *CD26* was among the six significantly upregulated genes in the NAWM (Fig. 3). A recent study also detected significant expression of *CD26* in both DNA methylation and RNA seq data in the NAWM tissue [33]. CD26/DPP4 is a membrane-associated exopeptidase that by engaging inhibitory ligands may limit autoimmunity in mice by regulating Th1 responses [65, 75], and by hydrolyzing substrates CXCL12 and CCL5 [12]. By using immunohistochemistry and immunofluorescence, we found that CD26 was expressed by microglia in the NAWM. In contrast, in active lesions, the morphology of CD26^+^ cells indicated lympho-monocytes rarely seen in the NAWM. *CD26* was significantly downregulated and CD26 protein expression was absent in chronic active lesions. These data suggested that CD26 may be related to an altered microglia function/phenotype in the NAWM that is absent in slowly expanding, chronic active lesions. The recent report of protection against cuprizone-induced demyelination by an inhibitory ligand of CD26 [18] also suggests regulation of microglia function, since the role of T cells in this model is probably minor [30, 67].

### The transcriptome signature and the distinctiveness of chronic active lesion

In order to investigate unique transcriptional changes at different stages of lesion evolution and fate, we applied a comprehensive approach: (i) we identified 62 signatures that were both differentially expressed and regulated at least among two lesion types; (ii) we extracted hundreds unique significant up- and downregulated genes in each lesion type, and created de novo enriched protein interaction networks with major hubs for these DEGs; (iii) we investigated predefined pathways based on DEGs that were present only in one lesion type.

The article "Unique RNA signature of different lesion types in the brain white matter in progressive multiple sclerosis" was retracted in 2019. Reasons: errors in the data; errors in the analysis; errors in the results or conclusions.

The global transcriptome heatmap of lesion evolution and fate was generated by a conservative approach: for each lesion type, genes had to be differentially expressed compared to the controls and they had to show at least three-fold different expression levels compared to at least one other lesion type. This analysis identified 62 DEGs with two clusters of genes with inverse regulation (Fig. 4). The heatmap of these genes indicated that chronic active lesion was the most different from all the other lesion types, and this difference was responsible for the inversely regulated two clusters. In addition, the signature of active lesions was more similar to inactive and remyelinating lesions than to chronic active lesions, suggesting a profound shift in molecular mechanisms underlying the active and chronic active lesion stage. The most different molecular signature was found between chronic active and remyelinating lesions.

Among the unique significantly upregulated genes specific to chronic active lesions, were the hypoxia-inducible transcription factor *ADM* gene [80] and the hypoxia-inducible protein *HILPDA* gene [58]. The cellular hypoxia and altered energy metabolism were also indicated by upregulation of genes related to energy metabolism (*ADSSL1, RBP7*), ion transport (*TRPV6, STC2*) and mitochondrial genes (*COX5BP6, GPD1*). These changes support the concept of virtual hypoxia, i.e. chronic oxidative injury associated with mitochondrial damage, demyelinated axons, and altered ion transport [1, 13, 16, 24, 56, 79]. Based on DEGs compared to control WM, energy metabolism pathways were under-represented in the MS-WM indicating a hypoxic state. Additionally, our data suggest that this hypoxic state is associated most with the chronic active lesions: these lesions exhibited the most DEGs for the mitochondrial respiratory chain and metabolic related genes among the top 100 up- and downregulated genes (29% in contrast to 12–16% in other lesion types). In addition, none of these DEGs (0%) in chronic active lesions were shared with the other lesion types, while 37–50% of such DEGs were shared by the active, inactive and remyelinating lesions. These data may indicate that chronic active lesions have the highest energy demand, mitochondrial and metabolic dysfunction. Genes of mitochondrial humanins (*MTRNR2L12, MTRNR2L8*) that may protect cells from oxidative stress [85] were significantly downregulated in chronic active lesions, while they were among the top 100 upregulated genes in active, inactive and remyelinating lesions. The gene of apoptosis inducing factor (AIF) that mediates caspase-independent death upon mitochondrial damage, and the gene of PARP1 that initiates this pathway in oligodendrocytes of MS lesions [81] were significantly downregulated in active, inactive and remyelinating MS lesions, while there was *PARP1* upregulation in chronic active lesions.

The article "Unique RNA signature of different lesion types in the brain white matter in progressive multiple sclerosis" was retracted in 2019. Reasons: errors in the data; errors in the analysis; errors in the results or conclusions.

Such overexpression of genes related to mitochondrial and energy failure was accompanied by gene enriched clusters related to focal adhesion, vascular smooth muscle contraction and ECM receptor interaction; all suggesting changes in the vasculature of chronic active lesions. This was not related to lymphocytic infiltrates, since perivascular CD20^+^ and CD3^+^ cells (*data not shown*) were exceptional, and inflammatory DEGs were scarce. The gene of the proangiogenic factor gene *VEGFA* and genes of extracellular matrix production (*GALNT6, ADAMTS14, TUBB4A*) were unique increased DEGs in chronic active lesions, while they were downregulated in the global MS-WM tissue, suggesting that vascular remodeling may be also a key player. This may compensate for the cellular hypoxia, or can be a primary alteration contributing to the hypoxic state. Such vascular molecular changes may add to the observed higher occurrence of vascular comorbidities in MS [78].

Other upregulated unique DEGs in chronic active lesions were related to negative regulation of neuronal growth (*ZNF536*), and inhibition of axonal outgrowth (*SEMA3B*). Such active inhibition of axonal growth in an increasing number of chronic active lesions can also contribute to the observed progressive loss of brain tissue [83].

Besides the upregulated cluster of unique DEGs in chronic active lesions, there was a cluster of unique downregulated DEGs, all upregulated in the other lesion types. One such gene was the growth hormone *IGF2*, indicating that remyelination potential and oligodendrocyte development is limited in chronic active vs other lesions. In line with our results, *IGF2* has been found downregulated in chronic active lesions [27] and increased in inactive lesions [86]. We also observed downregulation of *MERTK* in chronic active while upregulation in other lesion types. *MERTK* encodes for a member of the TAM family of tyrosine kinase receptors that are anti-apoptotic in oxidative stress conditions [6], mechanisms important in tissue repair. As MERTK inhibitors reduced myelin phagocytosis and induced proinflammatory cytokine response [69], the observed downregulation of *MERTK* could also contribute to the progressive tissue damage in chronic active lesion. Of note, MERTK was one the most upregulated genes in the global MS tissue compared to control, which also emphasize its selective downregulation in chronic active lesions. Other genes with inverse regulation also indicated reduced repair in chronic active lesions, i.e. downregulation of *FOXF1, FENDRR, PIK3R5, TNFRSF10D* and *GPNMB*.

The article "Unique RNA signature of different lesion types in the brain white matter in progressive multiple sclerosis" was retracted in 2019. Reasons: errors in the data; errors in the analysis; errors in the results or conclusions.

The de novo enriched protein interaction network of uniquely expressed DEGs in chronic active lesions contained two major hubs: the upregulated *IKBKG* gene coding for the NEMO protein (NF-kappa-B essential modulator) and the downregulated gene of N-cadherin (*CDH2*). Upregulation of NEMO that activates NF-κB may reflect ongoing innate immune responses and/or apoptosis in chronic active lesions. The downregulated major hub of *CDH2* with three other hubs of downregulated *PPRGC1A*, *DYRK1A* and *SLIT2* represented uniquely downregulated genes that participate in the generation of protective astrogliosis in response to CNS stress [2, 37, 39, 42, 63].

In conclusion, these data altogether indicate that the molecular mechanisms in chronic active lesions that are associated with development of secondary progression [16, 22, 39, 47, 62] are fundamentally different from the other lesion types. This also indicates that treatment considerations in the late phase of MS should be different from the earlier phases, when chronic active lesions are absent or less frequent. Particularly, treatment addressing the mitochondrial abnormalities and virtual hypoxia may be worth considering [44, 53, 76].

### Chitinase-3-like protein 1: expressed by astrocytes in the rim of chronic active lesions

We also found that *CHI3L1* was a unique upregulated DEG in chronic active lesions, while it was significantly downregulated in all other lesion types (Fig. 5). CHI3L1 (YKL-40) is a promising biomarker of inflammation in patients with progressive MS [71]. Immunohistochemistry and RNAscope proved the expression in chronic active lesions expressed in the rim primarily by astrocytes. Some previous data have suggested expression also by microglia beside astrocytes, in our samples both immunohistochemistry and combined RNAscope/immunohistochemistry indicated dominant expression by astrocytes [29]. These data suggest that some of the emerging biomarkers in progressive MS may reflect unique molecular changes in the brain related to specific lesion stages. The high expression of CHI3L1 in the CSF of patients with progressive MS [71] may be related to the increasing number of chronic active lesions, and we may speculate that its level in the CSF of patients with progressive MS may even reflect the number of chronic active lesions in the brain. The expression of CHI3L1 by astrocytes has been recently described in neurodegenerative diseases and often appears in clusters of astrocytes [48]. Knock-out animal models indicated a protective role of CHI3L1, as traumatic brain injury and experimental autoimmune encephalomyelitis were more severe in its absence [10, 82]. CH13L1 can influence the migratory capacity of astrocytes and reduces astrogliosis [10, 82]. CH13L1 can be induced in vitro by macrophages producing IL-1β, TNF-α and IL-6 [8, 10]. Despite the presence of macrophages/microglia close to CHI3L1 expressing cells in the rim in our study, genes of STAT3, IL-1β, TNF-α, and IL-6 were not significantly upregulated in chronic active lesions. Since *CHI3L1* was downregulated and the protein was not expressed either in other lesion types, astrocytic CHI3L1 may play a unique role in the pathogenesis of chronic active lesions: considering animal data [10, 82], it may dampen the inflammation and limit astrogliosis.

The article "Unique RNA signature of different lesion types in the brain white matter in progressive multiple sclerosis" was retracted in 2019. Reasons: errors in the data; errors in the analysis; errors in the results or conclusions.

### Remyelination versus chronic active lesions: de novo enriched network and TGFβ-R2

Observing the differences between chronic active and remyelinating lesions on the transcriptome heatmap (Fig. 4), we next examined those genes that were significantly but inversely regulated in these two lesion types, and created de novo networks based on protein interactions. The biggest network contained 62 genes upregulated in remyelinating lesions while downregulated in chronic active ones (Fig. 6). Upregulated genes of both pro-and anti-inflammatory molecules were represented in remyelinating lesions. Some of these molecules have been also indicated in reparatory processes, e.g. CXCL12 [64, 87]. Although we observed upregulated genes responsible for cell growth and DNA damage repair, myelin genes (MBP, MOG, PLP, MAG) were not upregulated. This was characteristic of all lesion types (*data not shown*) similar to recent data by microarray [86]. A very recent work that examined oligodendrocyte heterogeneity by single nuclei sequencing found that myelin-related genes were downregulated in OPCs of MS and NAWM, and the subclusters of mature oligodendrocytes were skewed between MS and control tissue [34]. The number of OPCs and oligodendrocytes are reduced in MS lesions [11, 34, 50], which may also be responsible for the observed absence of changes in myelin gene expression. Our additional analyses also supported repair in remyelinating lesions: (i) de novo network based on unique significant DEGs indicated several upregulated hubs related to oligodendrocyte genesis/myelination and cell growth regulation (*PDGFRA*, *CNTNAP2, TNR, EPS15, ANLN)*; (ii) the lesion signature heatmap also involved a number of genes initiating and supporting remyelination, regeneration, cellular growth, and anti-apoptosis (*IGF2, ADGRG6, CXCL12, MERTK, FOXF1, POK3R5, TNFRSF10D, GPNMB, MTRNR2L8, MTRNR2L12, KDR*). The absence of upregulated myelin genes may be related to the low number of oligodendrocytes in the lesions compared to control WM, and the heterogeneity of the incomplete remyelination stages in different lesions.

The article "Unique RNA signature of different lesion types in the brain white matter in progressive multiple sclerosis" was retracted in 2019. Reasons: errors in the data; errors in the analysis; errors in the results or conclusions.

The central hub in the de novo network of remyelinating versus chronic active lesions was TGFβ-R2 (Fig. 6). By immunohistochemistry and RNAscope, we found TGFβ-R2 expression by astrocytes in remyelinating lesions. A previous work detected TGFβ-R2 expression on hypertrophic astrocytes in chronic active lesions [25], but our transcriptome data suggested a strong downregulation of *TGFBR2* with FDR = 0.006 in such lesions. TGFβ has been associated with reparatory function in the CNS [15]. A recent bioinformatics study on microarray data from spinal cord periplaque vs. NAWM identified TGFβ1 in the context of astrocytosis and remodeling [59]. Astrocyte targeted overexpression of TGFβ1 resulted in earlier and more severe experimental autoimmune encephalomyelitis [52, 84], while systemic administration inhibited disease [43]. The effect of TGFβ in the CNS may depend on the lesion types that may exhibit different inflammatory and cellular environment including differential distribution of TGFβ receptors on different resident and infiltrating cells [15].

### Immunoglobulin genes

We noticed that immunoglobulin genes were among the top 10 upregulated genes in WM MS tissue vs. control WM (Fig. 7). The highly significant expression of immunoglobulin genes among the total MS-WM DEGs and especially in active and remyelinating lesions can be explained by presence of B cells, or by increased transcription of rearranged B cell receptors secreted also as antibodies. We detected the highest number of CD20^+^ B cells by immunohistochemistry in active lesions, but B cells were also present in remyelinating lesions. Studies have generally indicated that the WM lesions typically exhibit relatively few B cells and plasma cells in progressive MS [7, 47], and B cell-rich meningeal aggregates in the subpial cortical lesions are emphasized [49, 72, 73]. Here, we found B cells in WM lesions in at least 7 out of the 10 patients (Fig. 7c), and most of the B cells were detected in infiltrates around the vessels.

Some of the transcribed immunoglobulin genes may be secreted because among the top 10 upregulated is *J-CHAIN*, which serve to link immunoglobulins in dimer (IgA) or pentamer (IgM) as secretory components [35]. The dominance of immunoglobulin genes among the top upregulated DEGs was disproportional to the number of B cells, indicating either a restricted B cell clonality, or high secretion of immunoglobulins. When comparing the expression of immunoglobulin genes in different lesion types, we found the highest number and heterogeneity of upregulated variable region genes in remyelinating lesions, indicating that there may be a more heterogeneous B cell phenotype with paratopes to a wider range of epitopes in remyelinating lesions. Moreover, in remyelinating lesions we recognized the expression of *CD138*, a plasma cell marker [61] which further supports the presence of isotype switched matured B cells in remyelinating lesions besides CD20^+^ B cells, and this may be related to the most heterogeneous immunoglobulin gene repertoire. The role of B cells in remyelinating lesions were also emphasized by pathway analysis that detected upregulated B cell pathways. A recent work also emphasized the presence of plasma cells in lesions of patients with progressive MS [53]. Out of the seven detected heavy variable chain genes, three represented *IGHV4*. This transcript was also the most frequently found in B cell receptor transcriptome of the CSF and paired brain-draining lymph node tissue [36, 62, 76], and maybe related to rare T cell exposed motifs [31]. Altogether, these data argue for important role of B cells even in the WM of progressive MS. Whether the heterogeneous immunoglobulin genes in remyelinating lesions could reflect some special subset of B cells is not clear; we were not able to detect *IL10* transcripts in remyelinating lesions that may be related to regulatory B cells [74].

The article "Unique RNA signature of different lesion types in the brain white matter in progressive multiple sclerosis" was retracted in 2019. Reasons: errors in the data; errors in the analysis; errors in the results or conclusions.

## Conclusion

Our study is not without limitations. We used controls only without neurological disease. We did not separate rim and core in the chronic active and inactive lesions either. But the combination of different bioinformatics methods and validation by immunohistochemistry supported our conclusions, and such weakness does not hinder interpretation of changes in transcriptome signatures during lesion evolution and fate in the WM of progressive MS brain. Notable, the RNAscope validation on chronic active and remyelinating lesions from even the same patient confirmed that our results are not patient dependent but likely lesion dependent.

In conclusion, by next-generation RNA sequencing and a comprehensive computational systems medicine approach we identified mechanistic transcriptome signature of lesion evolution in the progressive MS brain WM. We found that the molecular signature of chronic active lesions was profoundly different from all other lesion types, and NAWM was more similar to control WM than to any other lesion types. It indicates that major gene expression changes occur both at early lesion genesis, and in lesions most characteristic as the late progressive phase develops. The highly specific mechanistic signature of chronic active lesions indicates that as these lesions develop in progressive MS, molecular pathways are substantially altered: the unique mitochondrial/metabolic changes and specific downregulation of molecules involved in tissue repair indicate a stage of exhaustion. Besides unique sub-networks mechanistically different at lesions stages, some molecules were specifically regulated: CD26/DPP4 upregulation by microglia in the NAWM suggesting that a special microglia subset characterized by CD26 may play a role in early lesion development; CH3L1 in the chronic active rim by astrocytes; TGFβ transcripts and TGFβ-R2 expressed by astrocytes in remyelinating lesions in contrast to lesions with chronic active tissue damage. The uniqueness of lesion types also indicates that omics approaches should consider lesion stages, when expression and regulation of different molecules are addressed. Although this study indicates the extreme diverse molecular events on transcriptome level at different lesion stages, yet our comprehensive unbiased search across subsets of multiple lesions provided a discovery of specific molecular mechanistic signatures validated by different approaches.

## Additional files

Additional file 1: **Table S1.** Clinical and demographic data of the MS patients and non-neurological disease controls (PDF 71 kb)

Additional file 2: Supplementary Methods (DOCX 49 kb)

Additional file 3: **Figure S1.** RNAscope: Negative (red and green targeting two bacterial genes) and positive (PPIB/POLR2A) controls. (PDF 320 kb)

Additional file 4: **Table S2.** Number of samples, detected genes and significant genes in the post-mortem human brain samples (PDF 181 kb)

Additional file 5: **Table S3.** Predefined pathways present based on the differentially expressed genes in each lesion type extracted from KEGG and GSEA (PDF 665 kb)

Additional file 6: **Table S4.** Differentially expressed genes related to oxidative stress, hypoxia and metabolic changes in the top 100 up- and downregulated genes of each lesion type (PDF 522 kb)

Additional file 7: **Figure S2.** Brain lesion prediction from Ingenuity Pathway Analysis (IPA) based on the genes with log2FC > 1 and FDR < 0.05 in the active lesions vs. WM control yellow = upregulated, blue = downregulated (PDF 2610 kb)

Additional file 8: **Table S5.** Top 10 up- and downregulated genes in lesion types vs control WM (PDF 262 kb)
